# A Combination Analysis of IVIM-DWI Biomarkers and T2WI-Based Texture Features for Tumor Differentiation Grade of Cervical Squamous Cell Carcinoma

**DOI:** 10.1155/2022/2837905

**Published:** 2022-03-17

**Authors:** Bin Shi, Jiang-Ning Dong, Li-Xiang Zhang, Cui-Ping Li, Fei Gao, Nai-Yu Li, Chuan-Bin Wang, Xin Fang, Pei-Pei Wang

**Affiliations:** ^1^Department of Radiology, The First Affiliated Hospital of USTC, Division of Life Sciences and Medicine, University of Science and Technology of China, Anhui Provincial Cancer Hospital, Hefei, 230031, China; ^2^Department of Radiology, The Third Affiliated Hospital of Xinxiang Medical College, Xinxiang, Henan 453003, China; ^3^Anhui Medical University, Hefei, Anhui 230000, China

## Abstract

**Purpose:**

To explore the value of intravoxel incoherent motion diffusion-weighted imaging (IVIM-DWI) and texture analysis on T2-weighted imaging (T2WI) for evaluating pathological differentiation of cervical squamous cell carcinoma.

**Method:**

This retrospective study included a total of 138 patients with pathologically confirmed poor/moderate/well-differentiated (71/49/18) who underwent conventional MRI and IVIM-DWI scans. The values of ADC, *D*, *D*^*∗*^, and *f* and 58 T2WI-based texture features (18 histogram features, 24 gray-level co-occurrence matrix features, and 16 gray-level run length matrix features) were obtained. Multiple comparison, correlation, and regression analyses were used.

**Results:**

For IVIM-DWI, the ADC, *D*, *D*^*∗*^, and *f* were significantly different among the three groups (*p* < 0.05). ADC, *D*, and *D*^*∗*^ were positively correlated with pathological differentiation (*r* = 0.262, 0.401, 0.401; *p* < 0.05), while the correlation was negative for *f* (*r* = −0.221; *p* < 0.05). The comparison of 52 parameters of texture analysis on T2WI reached statistically significant levels (*p* < 0.05). Multivariate logistic regression analysis incorporated significant IVIM-DWI, and texture features on T2WI showed good diagnostic performance both in the four differentiation groups (poorly vs. moderately, area under the curve(AUC) = 0.797; moderately vs. well, AUC = 0.954; poorly vs. moderately and well, AUC = 0.795; and well vs. moderately and poorly, AUC = 0.952). The AUCs of each parameters alone were smaller than that of each regression model (0.503∼0.684, 0.547∼0.805, 0.511∼0.712, and 0.636∼0.792, respectively; pairwise comparison of ROC curves between regression model and individual variables, *p* < 0.05).

**Conclusions:**

IVIM-DWI biomarkers and T2WI-based texture features had potential to evaluate the pathological differentiation of cervical squamous cell carcinoma. The combination of IVIM-DWI with texture analysis improved the predictive performance.

## 1. Introduction

Cervical carcinoma, as a malignant tumor in the female reproductive system, has a high incidence in China, and the increasing incidence and trend of younger age lead to a serious threat to health and life [1, 2]. The most common pathological type of cervical carcinoma is squamous cell carcinoma [3, 4], which can be divided into three grades of differentiation: poorly differentiated, moderately differentiated, and well-differentiated. Tumors at the early stage are mainly treated by surgery, while for patients with advanced tumors or those who need to preserve the uterus, radiation therapy may be chosen and is an effective method for cervical squamous cell carcinoma [5]. Some studies demonstrated that the tumor differentiation grade also has an impact on outcomes and survival [6]. Therefore, accurate radiological diagnosis for the prediction and evaluation of the pathological and molecular levels of cervical squamous cell carcinoma has been a hot topic in recent years, and many advanced techniques have been used in this area [7].

Intravoxel incoherent motion diffusion-weighted imaging (IVIM-DWI), as a noninvasive imaging tool, is able to distinguish the diffusion motion of water molecules and the perfusion-related contribution of the microcirculation system [7–9] and may provide more important cues to discover the correlation between radiology and pathology. The fine greyscale changes caused by the heterogeneity of lesions cannot be easily observed by traditional tools but can be measured by quantitative tools such as texture analysis [10]. For magnetic resonance imaging (MRI), T2-weighted imaging (T2WI) is highly sensitive to pathological processes because the characterization of the T2 signal allows for the determination of water content, degree of fibrotic change, necrosis, and haemorrhage in the tissue [11].

Therefore, our study aimed to explore the diagnostic value of IVIM-DWI and texture analysis on T2WI for the tumor differentiation grade of cervical squamous cell carcinoma. We hypothesized that the combination of IVIM-DWI biomarkers and texture features based on tumorous heterogeneity could develop a novel predictive paradigm for the formulation of operation or radiation therapy.

## 2. Materials and Methods

### 2.1. Patients

A total of 138 patients from our hospital with cervical squamous cell carcinoma between 2017 and 2020 were included in the study (Table 1). There were 71 patients in the poorly differentiated group, 49 patients in the moderately differentiated group, and 18 patients in the well-differentiated group. Differentiation was confirmed by pathology after surgery or biopsy.

The inclusion criteria of our study were as follows: (1) MRI routine examination was performed in our hospital within 2 weeks before any treatment; (2) no biopsy or therapy was performed before MRI examination; and (3) the image quality was adequate for diagnosis and measurement. The MRI scans and images could not reach the above criteria, such as the images have obvious motion artifacts, would be excluded in the study. This retrospective study was approved by our institutional review board with a waiver of written informed consent.

### 2.2. MRI Examination

All 138 patients underwent MRI examination by a 3.0 T MRI scanner (Signa HDxT, GE Healthcare, USA) equipped with an 8-channel phased array body coil. The patients lied in the supine position during the whole examination, including the conventional routine MRI sequences and IVIM-DWI for the assessment of the cervical lesions: (1) axial fast spin echo T1-weighted imaging (T1WI) of the pelvis (repetition time (TR) = 500 ms; echo time (TE) = 7.8 ms; thickness = 4 mm; and number of excitation (NEX) = 1); (2) sagittal and oblique (perpendicular to the long axis of the cervical canal) fast spin echo T2WI (TR = 4200 ms; TE = 68 ms; thickness = 4 mm; and NEX = 2); (3) axial fat-suppressed T2WI (TR = 4200 ms; TE = 68 ms; thickness = 4 mm; and NEX = 2); and (4) axial IVIM-DWI (TR = 4000 ms; TE = 77 ms; thickness = 4 mm; and NEX = 6; *b* = 0, 10, 20, 50, 100, 200, 400, 800, 1200 s/mm^2^). The whole acquisition time was 7 min and 54 s.

### 2.3. Image Acquisition

All original images in the DICOM format were divided into three groups depending on the tumor differentiation grade: poorly differentiated group, moderately differentiated group, and well-differentiated group. There were two parts of image analysis as described below (Figure 1).

#### 2.3.1. Part I: IVIM-DWI Measurement

Two radiologists (8 and 10 years of pelvic diagnostic experience, respectively) blinded to the pathological results and drew the region of interest (ROI) using the FuncTool software on a GE AW 4.6 postprocessing workstation. The ROI-1 of IVIM-DWI was selected on the maximum transverse plane of each lesion at *a b* value of 1200 s/mm^2^ to obtain the IVIM-DWI parameters of ADC, *D*, *D*^*∗*^, and *f*. For each case, the ROI-1 with 5 mm^2^ was drawn three times to acquire the average value, avoiding necrosis, haemorrhage, or cervical canal (each radiologist drew twice to get the values, and intraclass correlation coefficient was calculated to evaluate the interobserver agreement; Figure 2).

#### 2.3.2. Part II: Texture Analysis on T2WI

The ROI-2 was drawn on the oblique T2WI slice layer by layer to cover the whole tumor by using ITK-SNAP (version 3.6.0, http://www.itksnap.org) also in a blinded way. The two radiologists should reach an agreement on the chosen area of ROI-2. Considering that texture analysis should focus on the complete information of the lesions, ROI-2 was drawn on the whole lesion, including necrosis or haemorrhage inside (Figure 2). Then, 58 parameters of texture analysis were acquired by using a software package (Artificial Intelligence Kit version 3.2.2, GE Healthcare) (Table 2) [12].

### 2.4. Statistical Analysis

All quantitative variables above were analyzed by using SPSS version 22.0 and *G*^*∗*^ Power Version 3.1.9.2. The normality test and homogeneity test for variance were performed to explore the descriptive statistics. Depending on the results of normality test and homogeneity test for variance, we then chose one-way analysis of variance or nonparametric test to compare the difference for three groups. Pearson correlation analysis was used for the significant IVIM-DWI parameters. Then, depending on the test of parallel lines, we performed multivariate logistic regression to get the regression model of IVIM-DWI combined with texture features. Finally, the area under receiver operating characteristic (ROC) curves was used to assess the diagnostic value of regression models and each significant values. The sensitivity and specificity were also used to assess the combination of IVIM-DWI and texture features extracted on T2WI. In addition, statistical power analysis was used to evaluate the power value based on the total sample size in our study. *p* < 0.05 was selected as a significant level.

## 3. Results

### 3.1. Part I: IVIM-DWI Measurement

We used intraclass correlation coefficient to investigate the interobserver variability and found that the observers were in agreement on most of the IVIM-DWI parameters (0.881∼0.946, *p* < 0.05). The comparison of the ADC, *D*, *D*^*∗*^, and *f* values for tumor differentiation grade reached statistically significant levels (*p* < 0.05; Table 3). The ADC, *D*, and *D*^*∗*^ values were positively correlated with tumor differentiation grade (*r* = 0.262, 0.401, 0.401; *p* < 0.05 Figures 3(a)–3(c)), while the correlation between the *f* value and tumor differentiation grade was negative (*r* = −0.221; *p* < 0.05; Figure 3(d)).

### 3.2. Part II: Texture Analysis on T2WI

The comparison of 18 histogram features, 21 gray-level co-occurrence matrix features, and 13 gray-level run length matrix features reached statistically significant levels (*p* < 0.05, Figure 4). The comparison of cluster shade, inverse difference/ID, sum of squares, gray-level nonuniformity/GLN, run length nonuniformity/RLN, and run percentage/RP had no significant difference among three groups (*p* > 0.05).

The comparison of all pairwise significant variables indicated that: (1) most of the variables between the poorly and moderately differentiated groups had no difference (*p* > 0.05), but only the difference of inverse variance reached significant level (*p* < 0.05); (2) most of the variables between the poorly and well-differentiated groups and most of the variables between the moderately and well-differentiated groups were significant different (*p* < 0.05); and (3) the difference of skewness between the poorly and well-differentiated groups, and the range, joint entropy, IDM, LRE, and RV between the moderately and well-differentiated groups did not reach significant levels (*p* > 0.05).

### 3.3. Part III: Regression Analysis and Statistical Results of ROC

From the above analysis, there were 4 parameters of IVIM-DWI and 52 texture features on T2WI presented significant differences based on the tumor differentiation grade of cervical squamous cell carcinoma. After test of parallel lines, we used multivariate stepwise regression analysis to establish four regression models for differential diagnosis (poorly vs. moderately differentiated, moderately vs. well-differentiated, poorly vs. moderately and well-differentiated, well vs. moderately and poorly differentiated; *p* < 0.05, Table 4). According to the ROC curves, the areas under the curve (AUC) of these regression model for four comparison were 0.797, 0.954, 0.795, and 0.952, respectively (Table 4, Figure 5); better than each parameters of IVIM-DWI and texture features on T2WI alone (0.503∼0.684, 0.547∼0.805, 0.511∼0.712, and 0.636∼0.792, respectively); all pairwise comparison of ROC curves between regression model and individual variables reached *p* < 0.05. The sensitivities and specificities of the four regression models are listed in Table 4.

The statistical power analysis revealed that the statistical power value (1-*β* error probability) of regression analysis was 0.99 based on our total sample size of 138 and given an *α* error probability of 0.05.

## 4. Discussion

### 4.1. The Diagnostic Performance of IVIM-DWI

The conventional diagnosis of cervical carcinoma and its clinical stage mainly depend on the morphological characteristics of lesions and the clinical experiences of radiologists [13]. Recently, with the improvement of radiological techniques, especially in MRI, doctors could obtain more information to further assess the disease and make more accurate decisions for individual treatment strategies [14]. Diffusion-weighted imaging (DWI) can reflect the diffusion motion of water molecules in tissues [15]. IVIM-DWI using multiple *b* values and a biexponential model could calculate not only the ADC value to reflect the combination of the diffusion and perfusion information of the tumor tissues and biological conditions but also the *D* value to represent the pure diffusion motion of water molecules, the *D*^*∗*^ value to represent the perfusion of the microcirculation, and the *f* value to represent the volume of blood flowing into the capillary [16].

Cervical squamous cell carcinoma mainly occurs at the junction of the cervix squamous and columnar epithelium [17]. With the decrease in tumor differentiation grade, more obvious atypia of tumor cells, less cytoplasm, and a higher cytoplasmic ratio could be observed by microscopy, indicating more malignant tumors [18]. According to our study, the differences in the ADC, *D*, *D*^*∗*^, and *f* values among the groups of poorly differentiated, moderately differentiated, and well-differentiated cases reached statistically significant levels (*p* < 0.05). Although the malignant squamous cells in the tumors were mainly arranged in solid cancer nests and the central keratin protein structure was tight [18], our study still found important evidence to differentiate the three groups.

Based on the results of correlation analysis, we found that the ADC, *D*, and *D*^*∗*^ values were positively correlated with tumor differentiation grade (*r* = 0.262, 0.401, 0.401; *p* < 0.05), while the correlation between the *f* value and tumor differentiation grade was negative (*r* = −0.221; *p* < 0.05). First, lesions with poorer differentiated and a higher malignant tendency had smaller *D* values, which meant that the water molecules in the lesions were restricted more than those in higher differentiated lesions, similar to the findings of other studies of malignancies [19, 20]. Second, smaller *D*^*∗*^ values were seen in poorly differentiated, indicating that the blood flow in the microcirculation would be more limited by the vessel wall or influenced by the fluid viscosity. Cancer cells invade the vessels and produce emboli, which would impact the blood flow, and these events could be observed more in tumors with poorer differentiated. Previous studies have shown that malignant tissues yield lower diffusion and perfusion characteristics than normal tissues [21, 22], as reflected by the positive correlation between the *D* and *D*^*∗*^ values and tumor differentiation grade. Third, the ADC value reflects the information of both water molecules and microcirculation. Fourth, the *f* value was negatively correlated with tumor differentiation grade. In our study, the negative tendency with tumor differentiation grade was similar to the *f* value because the *f* value was affected by T2 contribution [23]. The results showed that lesions with poorer differentiated had a more abundant blood supply for the tumor. Therefore, the proportion of perfusion-related contributions was also higher.

In our study, we chose 9 *b* values, 6 of which were less than 200 s/mm^2^ to improve the consistency and stability of the results, as shown in a previous study [24, 25]. Therefore, the study showed that IVIM-DWI had the ability to investigate microscopic changes in complex biological conditions and is worthy of consolidation and exploration.

### 4.2. The Diagnostic Performance of Texture Features on T2WI

Texture analysis is an advanced tool to objectively and quantitatively obtain the texture features of the heterogeneity within a lesion by taking into account pixel intensity, spatial location, and relationship of pixels in the image [26]. Some studies revealed that texture analysis has effective differential diagnostic performance on a variety of lesions [27, 28]. In the study, we chose the lesions on T2WI to acquire the texture features according to the high sensitivity to pathological changes of this sequence [11]. The characterization of the T2 signal depends on the lesions and the pathological changes such as fibrosis, necrosis, or haemorrhage inside. With texture analysis, we could not only discover the slight changes of lesions which cannot be easily observed by radiologist but also measure the greyscale changes in quantitative way.

In pairwise analysis, we could conclude that the texture features on T2WI helped the differential diagnosis of tumor differentiation grade of cervical squamous cell carcinoma, especially for the well vs. poorly/moderately differentiated groups. The texture features could improve our understanding on the heterogeneity of lesions with tumor differentiation grade (Table 2) [12]. In discussion, we highlighted the five texture features accepted in the establishing of regression model. They were range, IDMN, inverse variance, difference average, and SRHGLE.

The difference of range, IDMN, inverse variance, difference average, and SRHGLE in poorly vs. moderately differentiated lesions was similar, which meant the range of gray values, homogeneity, regular degree of texture, the relationship between occurrences of pairs with similar intensity values, and occurrences of pairs with differing intensity values, and the joint distribution of shorter run lengths with higher gray-level values were similar in these two groups.

The range of poorly or moderately differentiated lesions was significantly larger than that of well-differentiated groups, indicating that the lesions with poorer differentiation had larger intensity on T2WI [9]. The appearance of IDMN implied that the lesions with poorly differentiated had greater heterogeneity by evaluating the homogeneity [12]. The difference of these two features supported that the poorly differentiated cervical squamous cell carcinoma manifests with necrosis or haemorrhage more often [6]. The parameter of inverse variance described the regular degree of the texture [9], confirming the lesions with well-differentiated seemed to have more regular texture and a poorer visual effect. The difference average of poorly or moderately differentiated groups were significant smaller than that of well-differentiated group. Difference Average measures the relationship between occurrences of pairs with similar intensity values and occurrences of pairs with differing intensity values [12], supporting the tumor heterogeneity was more obvious with lower pathological differentiation. SRHGLE is one of the features of gray-level run length matrix and quantifies gray-level runs, which are defined as the joint distribution of shorter run lengths with higher gray-level values [12]. The SRHGLE of poorly or moderately differentiated lesions were significant smaller than that of well-differentiated lesions, implying that the lesions with higher differentiated had more fine textural textures and a greater concentration of high gray-level values in the images.

### 4.3. The Combination of IVIM-DWI and Texture Analysis

Finally, we carried out a combined analysis of IVIM-DWI and T2WI-based texture analysis. We hypothesized four compared groups for regression analysis (Table 4). According to the ROC curves, the AUCs of these regression model for four comparison were 0.797, 0.954, 0.795, amd 0.952, respectively; better than each parameters of IVIM-DWI and texture features on T2WI alone (0.503∼0.684, 0.547∼0.805, 0.511∼0.712, and 0.636∼0.792, respectively). Then, we concluded that the regression models we built could study diffusion, perfusion, and tumor heterogeneity information in a comprehensive way. Since the tumor differentiation grade has an impact on outcomes and survival [6], by using IVIM-DWI and texture analysis on T2WI together, researchers can establish an imaging-based model related to the microcirculation system and tumor heterogeneity, to further acknowledge the disease and make more accurate decisions for treatment strategies.

The limitations of the study included are as follows: first, the number of well-differentiated groups in the retrospective study was relatively small (only 18 cases), increasing the risk of bias; second, in our study, ROI of image segmentation was performed manually, which may be influenced by the subjective or objective factors of interobserver and intraobserver variability.

## 5. Conclusion

IVIM-DWI biomarkers and T2WI-based texture features had potential to evaluate the pathological differentiation of cervical squamous cell carcinoma. The combination of IVIM-DWI with texture analysis improved the predictive performance. The performance of the effective imaging-based tools was closely associated with the pathological basis, which might be helpful to make up for the deficiency of biopsy, to develop scientific and individualized treatment, and to further improve prognosis in the clinical process.

## Figures and Tables

**Figure 1:** The steps of image acquisition and statistical analysis.

**Figure 2:** Examples of manually drawing ROIs for cervical squamous cell carcinoma. Panels A–H belong to a 50-year-old female with cervical squamous cell carcinoma of well-differentiated. On panel A (IVIM-DWI at 1200 s/mm^2^), each radiologist drew ROI-1 (5 mm^2^) three times to get the values on the maps of ADC, *D*, *D*^*∗*^, and *f*, respectively (panels B–E). Panel F is the maximum area of the lesion on T2WI, so the radiologist drew ROI-2 of the whole lesion on panel G. Panel H is the pathological performance, HE *∗* 400.

**Figure 3:** Correlation results of IVIM-DWI based on degree of differentiation. Panels A∼D are the tendencies of the correlation between ADC, *D*, *D*^*∗*^, *f* values and pathological differentiation visualized by scatter diagrams. The labels “0,” “1,” and “2” represent the poorly, moderately, and well-differentiated groups, respectively.

**Figure 4:** Statistical results of multiple comparison analysis of texture features on T2WI. Panels A∼C are the column diagrams of significant texture features (*p* < 0.05). The red, yellow, and green column represent the poorly, moderately, and well-differentiated groups, respectively. The abbreviations are listed in Table 2.

**Figure 5:** Statistical results of ROC curves.

**Table 1:** The basic information of patients and lesions in this study.

Group/*p* value	*n* ^a^	Age	Length of lesions	Number of surgery/biopsy
Poorly differentiated	71	51.37 ± 9.95 (range: 27∼78)	26.92 ± 8.48	36/35
Moderately differentiated	49	51.98 ± 9.84 (range: 31∼73)	28.36 ± 9.73	28/21
Well-differentiated	18	54.56 ± 11.83 (range: 38∼88)	27.67 ± 7.39	7/11
*p* value ^*b*^	—	0.495^c^	0.677^c^	0.409^d^

^a^Number of cases in each group. ^b^Statistically significant difference (*p* < 0.05). ^c^Analysis of variance. ^d^Pearson chi-square test. The parameters of age and length of lesions with normal distributions are presented as the mean ± standard deviation.

**Table 2:** The parameters of texture analysis used in this study.

Methods	Features	Number of features
Histogram	Energy, total energy, entropy, minimum, 10th percentile, 90th percentile, maximum, mean, median, interquartile range, range, mean absolute deviation (MAD), robust mean absolute deviation (rMAD), root mean squared (RMS), skewness, kurtosis, variance, uniformity	18
Gray-level co-occurrence matrix (GLCM)	Autocorrelation, joint average, cluster prominence, cluster shade, cluster tendency, contrast, correlation, difference average, difference entropy, difference variance, joint energy, joint entropy, informational measure of correlation (IMC) 1, informational measure of correlation (IMC) 2, inverse difference moment (IDM), maximal correlation coefficient (MCC), inverse difference moment normalized (IDMN), inverse difference (ID), inverse difference normalized (IDN), inverse variance, maximum probability, sum average, sum entropy, sum of squares	24
Gray-level run length matrix (GLRLM)	Short run emphasis (SRE), long run emphasis (LRE), gray-level nonuniformity (GLN), gray-level nonuniformity normalized (GLNN), run length non-uniformity (RLN), run length non-uniformity normalized (RLNN), run percentage (RP), gray-level variance (GLV), run variance (RV), run entropy (RE), low gray-level run emphasis (LGLRE), high gray-level run emphasis (HGLRE), short run low gray-level emphasis (SRLGLE), short run high gray-level emphasis (SRHGLE), long run low gray-level emphasis (LRLGLE), long run high gray-level emphasis (LRHGLE)	16

**Table 3:** The comparison of IVIM-DWI parameters.

Group/*p* value	*n* ^a^	ADC	*D*	*D* ^*∗*^	*f*
Poorly differentiated	71	0.74 ± 0.10	0.54 (0.16)	9.13 (11.10)	29.50 (24.80)
Moderately differentiated	49	0.79 ± 0.14	0.63 ± 0.10	17.30 (9.93)	22.60 (5.92)
Well-differentiated	18	0.82 ± 0.12	0.73 ± 0.13	31.32 ± 16.95	18.80 (6.43)
*p* value^*b*^	—	0.006	<0.001	<0.001	0.034

^a^Number of cases in each group. ^b^Statistically significant difference (*p* < 0.05). The units of the ADC, *D*, and *D*^*∗*^ values are ^*∗*^10^−3^ mm^2^/s, and the unit of the *f* value is %. The parameters with normal distributions are presented as the mean ± standard deviation, and the parameters with skewed distributions are presented as the median (interquartile range). The analysis of variance was used for the ADC value, and the nonparametric test was used for *D*, *D*^*∗*^, and *f* values.

**Table 4:** Statistical results of regression analysis.

	Regression model	AUC (95% CI)	Sensitivity	Specificity
Poorly vs. moderately	*Ŷ* = 30.43 − 6.755 *∗* *f* − 2.772 *∗* difference average − 50.441 *∗* inverse variance − 0.007 *∗* SRHGLE	0.797 (0.718–0.875)	97.96	50.70
Moderately vs. well	*Ŷ* = 13.918–23.142 *∗* ADC + 22.326 *∗* *D* + 0.08 *∗* *D*^*∗*^ − 15.405 *∗* IDMN	0.954 (0.882–1.000)	93.88	94.44
Poorly vs. moderately and well	*Ŷ* = 1.486 + 3.903 *∗* *D* − 5.558 *∗* *f* − 0.003 *∗* range	0.795 (0.720–0.870)	88.06	64.79
Well vs. moderately and poorly	*Ŷ* = 14.644–30.501 *∗* ADC + 33.041 *∗* *D* − 16.553 *∗* IDMN	0.952 (0.888–0.952)	91.69	94.44

IDMN represented for inverse difference moment normalized. SRHGLE represented for short run high gray-level emphasis. The units of the sensitivity and specificity are %.

## Data Availability

The raw data supporting the conclusions of this article will be made available by the authors, without undue reservation.

## References

[1] Balleyguier C., Sala E., Da Cunha T. (2011). Staging of uterine cervical cancer with MRI: guidelines of the European Society of Urogenital Radiology. *European Radiology*.

[2] Burzawa J., Gonzales N., Frumovitz M. (2015). Challenges in the diagnosis and management of cervical neuroendocrine carcinoma. *Expert Review of Anticancer Therapy*.

[3] Vinh-Hung V., Bourgain C., Vlastos G. (2007). Prognostic value of histopathology and trends in cervical cancer: a SEER population study. *BMC Cancer*.

[4] Bhatla N., Aoki D., Sharma D. N., Sankaranarayanan R. (2018). Cancer of the cervix uteri. *International Journal of Gynecology & Obstetrics*.

[5] FIGO Committee on Gynecologic Oncology (2014). FIGO staging for carcinoma of the vulva, cervix, and corpus uteri. *International Journal of Gynaecology & Obstetrics*.

[6] Matsuo K., Mandelbaum R. S., Machida H. (2018). Association of tumor differentiation grade and survival of women with squamous cell carcinoma of the uterine cervix. *Journal of gynecologic oncology*.

[7] Jonska-Gmyrek J., Gmyrek L., Zolciak-Siwinska A., Kowalska M., Kotowicz B. (2019). Adenocarcinoma histology is a poor prognostic factor in locally advanced cervical cancer. *Current Medical Research and Opinion*.

[8] Thapa D., Wang P., Wu G., Wang X., Sun Q. (2019). A histogram analysis of diffusion and perfusion features of cervical cancer based on intravoxel incoherent motion magnetic resonance imaging. *Magnetic Resonance Imaging*.

[9] Le Bihan D., Breton E., Lallemand D., Aubin M. L., Vignaud J., Laval-Jeantet M. (1988). Separation of diffusion and perfusion in intravoxel incoherent motion MR imaging. *Radiology*.

[10] Zhang S., Chiang G. C.-Y., Magge R. S. (2019). MRI based texture analysis to classify low grade gliomas into astrocytoma and 1p/19q codeleted oligodendroglioma. *Magnetic Resonance Imaging*.

[11] Dushyant V. S., Anthony E. S. (2011). *Abdominal Imaging*.

[12] Zwanenburg A., Leger S., Vallières M., Löck S. (2019). Image biomarker standardisation initiative. https://arxiv.org/pdf/1612.07003.pdf.

[13] Cornelis F., Tricaud E., Lasserre A. S. (2014). Routinely performed multiparametric magnetic resonance imaging helps to differentiate common subtypes of renal tumours. *European Radiology*.

[14] Wakefield J. C., Downey K., Kyriazi S., deSouza N. M. (2013). New MR techniques in gynecologic cancer. *American Journal of Roentgenology*.

[15] Lin Y., Li H., Chen Z. (2015). Correlation of histogram analysis of apparent diffusion coefficient with uterine cervical pathologic finding. *American Journal of Roentgenology*.

[16] Le Bihan D., Breton E., Lallemand D., Grenier P., Cabanis E., Laval-Jeantet M. (1986). MR imaging of intravoxel incoherent motions: application to diffusion and perfusion in neurologic disorders. *Radiology*.

[17] Doorbar J., Griffin H. (2019). Refining our understanding of cervical neoplasia and its cellular origins. *Papillomavirus Research*.

[18] Fatteneh A., Tavassoli P. D. (2003). *Pathology and Genetics of Tumours of the Breast and Female Genital Organs*.

[19] Winfield J. M., Orton M. R., Collins D. J. (2017). Separation of type and grade in cervical tumours using non-mono-exponential models of diffusion-weighted MRI. *European Radiology*.

[20] Zhou Y., Liu J., Liu C. (2016). Intravoxel incoherent motion diffusion weighted MRI of cervical cancer - correlated with tumor differentiation and perfusion. *Magnetic Resonance Imaging*.

[21] Koh D.-M., Collins D. J., Orton M. R. (2011). Intravoxel incoherent motion in body diffusion-weighted MRI: Reality and challenges. *American Journal of Roentgenology*.

[22] Lee E. Y. P., Yu X., Chu M. M. Y. (2014). Perfusion and diffusion characteristics of cervical cancer based on intraxovel incoherent motion MR imaging-a pilot study. *European Radiology*.

[23] Bashir U., Siddique M. M., Mclean E., Goh V., Cook G. J. (2016). Imaging heterogeneity in lung cancer: techniques, applications, and challenges. *American Journal of Roentgenology*.

[24] Fournet G., Li J.-R., Cerjanic A. M., Sutton B. P., Ciobanu L., Le Bihan D. (2017). A two-pool model to describe the IVIM cerebral perfusion. *Journal of Cerebral Blood Flow and Metabolism*.

[25] Wan Q., Deng Y. S., Zhou J. X. (2017). Intravoxel incoherent motion diffusion weighted MR imaging in assessing and characterizing solitary pulmonary lesions. *Nat Publ Group*.

[26] Su C.-Q., Lu S.-S., Zhou M.-D., Shen H., Shi H.-B., Hong X.-N. (2019). Combined texture analysis of diffusion-weighted imaging with conventional MRI for non-invasive assessment of IDH1 mutation in anaplastic gliomas. *Clinical Radiology*.

[27] Kumar V., Gu Y., Basu S. (2012). Radiomics: the process and the challenges. *Magnetic resonance imaging*.

[28] Liu J., Wan Y., Wang Z., Qi Y., Qu P., Liu Y. (2016). Perfusion and diffusion characteristics of endometrial malignancy based on intravoxel incoherent motion MRI at 3.0 T: comparison with normal endometrium. *Acta Radiologica*.

